# A Novel Method for Remaining Useful Life Prediction of Roller Bearings Involving the Discrepancy and Similarity of Degradation Trajectories

**DOI:** 10.1155/2021/2500997

**Published:** 2021-12-02

**Authors:** Honglin Luo, Lin Bo, Xiaofeng Liu, Hong Zhang

**Affiliations:** The State Key Laboratory of Mechanical Transmission, Chongqing University, Chongqing 400044, China

## Abstract

Accurate remaining useful life (RUL) prediction of bearings is the key to effective decision-making for predictive maintenance (PdM) of rotating machinery. However, the individual heterogeneity and different working conditions of bearings make the degradation trajectories of bearings different, resulting in the mismatch between the RUL prediction model established by the full-life training bearing and the testing bearings. To address this challenge, this paper proposes a novel RUL prediction method for roller bearings that considers the difference and similarity of degradation trajectories. In this method, a feature extraction method based on continuous wavelet transform (CWT) and convolutional autoencoder (CAE) is proposed to extract the deep features associated with bearing performance degradation before the degradation indicator (DI) is obtained by applying the self-organizing maps (SOM) method. Next, a dynamic time warping (DTW) based method is applied to perform the similarity matching of degradation trajectories of the training and testing bearings. Driven by the historical DIs of the given bearing, the grey forecasting model with full-order time power terms (FOTP-GM) is applied to model the degradation trajectory using a parameter optimization method. Then, the failure threshold of the given testing bearing can be determined using a data-driven method without manual intervention. Finally, the RUL of the given testing bearing can be estimated using the preset failure threshold and the optimized degradation trajectory model of the given testing bearing. The experimental results show that the proposed method retains the individual differences of bearing degradation trend, realizes the independent and reasonable bearing failure threshold setting, and improves the prediction accuracy of RUL.

## 1. Introduction

Accurate remaining useful life (RUL) estimation of bearings is a significant challenge in the prognostics and health management (PHM) system for rotating machinery to improve the equipment reliability and reduce equipment failures as well as maintenance costs. In the literature, the prognostic approaches in a PHM framework can be implemented in three different ways: physics-based approaches, data-driven approaches, and hybrid approaches (a combination of data-driven and physics-based approaches) [1]. By solving a set of equations based on the physical laws and the knowledge of engineering and science, the physics-based prognostic approaches assess the component health and predict when the damage crosses a predefined failure threshold based on the mathematical modeling of the degradation process for a particular failure mode [2]. However, with high accuracy and efficiency requirements in component RUL prediction, physical model-based life prediction methods are difficult to meet modern needs due to their complexity, time-consuming, and nonuniversality.

Without considering the complex degradation mechanism of the system, the data-driven-based prognostic approaches can reduce the dependence on the amount of prior knowledge and have the advantages of high prediction accuracy and strong applicability. From the perspective of mathematical modeling, the data-driven prognostic methods can be further divided into statistical methods and artificial intelligence (AI) based methods [3]. Statistics-based prognostic approaches, also known as the empirical model-based prognostic approaches, estimate the remaining useful life of a mechanical component by building a statistical model based on empirical knowledge. The statistical methods include Gaussian model methods, autoregressive model methods, hidden Markov model (HMM) methods, Wiener process model methods, various statistical clustering methods based on distance, and so on. Medjaher et al. [4] proposed a mixture bearing RUL prediction model combining the Gaussian model and HMM, and the performance of the proposed method is verified using the real degradation data sets of bearings. C. Kwan et al. [5] proposed a novel bearing fault diagnostics and prognostics method using HMM to characterize the failure mechanism of bearings and applied the HMM-based method to a rotating shaft system to verify its performance using actual data. X. Zhang et al. [6] proposed an integrated method for bearing fault diagnostic and prognostic based on PCA and HMM, and the effectiveness of the proposed method is verified by using experimental bearing vibration data sets. P. Ding et al. [7] proposed a novel degradation trend estimation method based on an interpretable and lightweight vector autoregression algorithm, and the run-to-failure data sets of rolling and slewing bearings are analyzed to demonstrate the effectiveness of the proposed method. B. Ayhan et al. [8] proposed an adaptive bearing RUL prediction method based on the damage accumulation description, in which the recursive least squares (RLS) algorithm is applied to estimate the damage curve approach (DCA) based RUL prediction model adaptively.

The main way to perform an AI-based framework for bearing RUL prediction is machine learning (ML) based prognostics, including artificial neural networks (ANN) [9], support vector machines (SVM) [10], random forests (RF) [11], and deep learning (DL) [12]. The conventional machine learning-based prognostic methods usually extract a single statistical feature in time or frequency domain from the original signal as a health index (HI), such as root mean square [13], Kurtosis [14], energy entropy [15], and so on. However, there are significant limitations in the characterization capability of such single statistical features. To a more reasonable degradation indicator (DI), different statistical features are extracted in time, frequency, and time-frequency domain, and some DI construction methods, such as the principal component analysis (PCA) [16], support vector data description (SVDD) [17], self-organizing map (SOM) [18], and orthogonal sparse algorithm (OSA) [19], are applied to fuse an effective degradation indicator by reducing the dimension of such extracted feature sets.

The deep-learning-based prognostic methods can learn the deep information of original data and accurately evaluate the degradation status of bearings. The deep-learning-based methods applied to predict the bearing RUL mainly include: deep belief networks (DBN) [20], integrated deep learning method based on time domain and frequency domain features [21], convolutional neural network (CNN) [22,23], autoencoder (AE) [24], recurrent neural network (RNN) [25], and long short-term memory (LSTM) [26]. It should be noted that the deep learning methods mentioned above usually use the full-life-cycle data of the training bearing to build a deep learning model to establish a nonlinear mapping relationship between the monitoring data of testing bearing and its RUL under the assumption that the degradation patterns of the training bearing and the test bearing are the same or similar. In practical engineering practice, due to the individual heterogeneity of bearings and different environmental conditions, bearings under the same working condition may not necessarily have similar degradation trajectories, while bearings under different working conditions may also have similar degradation trends. In addition, a sufficient volume of bearings with full-life data is needed as a prerequisite to training a practicable prediction model using deep learning methods, but it is not easy to collect large amounts of bearing data with health information marked since the collection of bearing data is complex and expensive.

To address the mismatch between the pretrained RUL prediction model and the test bearing, one approach is to map the pretrained model or the testing data by employing transfer learning (TL) approaches to adapt the prediction model to the test bearing domain [27]. To this end, many researchers have extensively explored transfer learning methods, such as transfer component analysis (TCA) [28], joint distribution adaptation (JDA) [29], and correlation alignment (CORAL) [30]. Aiming at bearing RUL prediction based on transfer learning, Mao et al. [31] adopted TCA to bridge the RUL discrepancy between test bearings and training bearings. P. Ding et al. [32] proposed a novel bearing RUL assessment method based on unsupervised meta-learning to deal with the challenge of poor generalization and low prediction accuracy resulting from unlabelled and limited samples. Y. Ding et al. [33] proposed a dynamic domain adaptation-based RUL prediction method for the machinery with multiple working conditions using a deep subdomain adaptive regression network. X. Li et al. [34] proposed a deep learning-based prognostic method in which the generative adversarial network is used to learn the distribution of the healthy state data. However, it is worth noting that it is a time-consuming task with a tremendous computational burden to perform the transfer learning for high RUL predicting accuracy. Besides, the nonlinear relationship between the training data and the RUL prediction model after domain adaptation is not necessarily suitable for all the target test bearing data sets due to the individual heterogeneity of the bearings.

Another approach for cross-domain RUL prediction problems is the degradation indicator extrapolation method. The DI extrapolation method sets a reasonable failure threshold according to the data characteristics of the given test bearing, then establishes a fitted degradation model of the test bearing according to its historical DI curve, and finally realizes the RUL prediction of the given testing bearing based on the preset failure threshold and fitted the DI curve. Compared to the black-box transfer learning-based methods, the DI extrapolation method has good physical interpretability. The challenges in this method are how to fit the bearing historical DI curve quickly and accurately and how to determine the failure threshold automatically with no human intervention, in which three issues should be addressed carefully:

1. Building a degradation model for the given bearing using practical features that can characterize the performance degradation of bearing
2. Setting practicable failure thresholds for the testing bearings with different performance degradation patterns
3. Establishing a prediction framework with a good generalization ability that can update the model parameters dynamically according to bearing test information

As an approximate exponential model, the grey forecasting model (GM) can analyze the internal law of the grey system with fuzzy structure and incomplete or uncertain exponential data, showing a high forecasting precision and robust performance. K. Peng et al. [35] proposed an aircraft engine RUL method using GM (1, 1) model with a better RUL prediction performance by taking logarithmic operations and sliding window prediction. Z. Meng et al. [36] combines the Markov and GM (1, 1) models to realize the bearing RUL prediction, showing a lower root mean square percentage error. Note that the traditional grey models cannot simulate accurately any given nonhomogeneous exponential sequence with velocity and acceleration terms, a novel grey forecasting model with full-order time power terms (FOTP-GM (1, 1)) is proposed to solve this problem by S. Li et al. [37]. The FOTO-GM (1, 1) model can simulate a more complex approximate exponential sequence containing constant, velocity, and acceleration terms by changing its structure automatically to adapt to the evolution trend of parameters to be predicted. The FOTO-GM (1, 1) model can fit the homogeneous exponential sequence exactly and simulate such nonhomogeneous exponential, which provides another new approach for grey theory in bearing RUL prediction.

The accuracy of bearing RUL prediction is not only affected by the bearing degradation model but also closely related to the failure threshold. A reasonable failure threshold can make the facility managers carry out more effective maintenance depending on the bearing health condition. In the existing literature on data-driven based bearing RUL prediction, there are few discussions on the setting of failure threshold, and most of them are set manually, which mainly includes four setting methods: manual empirical method [38], vibration acceleration amplitude threshold of 20 g [31], and life percentage uniform threshold [39]. These failure threshold setting methods have a significant manual subjectivity and do not consider the variability of the bearing performance degradation process, and their engineering utility is limited. In the engineering practice, the degradation trends of bearings under the same working conditions may be different, while the degradation trends of bearings under different working conditions are similar to some extent due to individual heterogeneity and different environmental conditions of bearings. Therefore, the difference and similarity of the degradation trends between the training and test bearings must be taken into account when performing the bearing RUL prediction.

Some researches have been done to fill this gap. Wang *T* et al. [40] proposed a novel RUL prediction method based on the degradation trajectory similarity using the Euclidean distance as the similarity criterion, and the smaller the distance, the greater the similarity. Li et al. [41] proposed a similarity-based approach for RUL estimation for industrial components by calculating the fuzzy similarity between test trajectory patterns and reference training trajectory patterns. However, the similarity measure methods mentioned above need to unify the sequence length using the average method or the interpolation method resulting in the loss of the original time information of the degradation trajectories. Dynamic time warping [42], which can effectively cluster time series with noise and time distortion, is an effective pattern dissimilarity measurement technique that can align two different length sequences representing the same type of things in the time domain and calculate the distance between the two-time series by extending and shortening the time series.

Given the challenges and discussion above, this work proposes a bearing RUL prediction approach that considers the difference and similarity of bearing degradation trajectories. In the proposed method, the DTW is used to measure the similarities between degradation trajectories of the training and testing bearings, and the FOTO-GM (1, 1) model is utilized to fit the degradation trajectory of the given bearing with high simulative precision. Firstly, the time-frequency diagrams of the training and testing bearings are generated by CWT before the deep features associated with the performance degradation are extracted by inputting such time-frequency representations into the CAE network. Secondly, the degradation trajectories of the training and testing bearings can be obtained by inputting such hidden features into the pretrained SOM networks. Then, the fitted degradation trajectories models of the training and testing bearings are obtained by the FOTO-GM (1, 1) model, and the failure thresholds of testing bearings can be determined using the fitted degradation curves of the training bearings and the degradation trend distances between the training and testing bearings measured by DTW. Finally, the RUL prediction of the testing bearings can be realized using the preset failure thresholds and fitted degradation curves of testing bearings.

The proposed framework is evaluated on the IEEE PHM 2012 Challenge data sets [43] and the XJTU-SY data sets [44]. The case study on experimental bearing data sets proves that the proposed method could accurately predict the RUL of bearings under different working conditions. The comparison with other state-of-the-art methods also verifies the feasibility of the proposed method. The main contributions of this paper are summarized as follows:

1. A CWT-CAE-SOM-based bearing degradation indicator construction method is proposed without manual steps of signal feature extraction, selection, and fusion. This method extracts the hidden deep representations driven by the monitoring data of the given bearing to meet the consideration of the difference and independence between the full-life training bearing and test bearings. Then the DI can be obtained using the SOM network pretrained by the normal state deep features without considering the influence of the insufficient degradation data of the test bearing.
2. A DTW-based bearing degradation trend similarity matching method is proposed. This method calculates the DTW distances between historical degradation trajectories of the training and testing bearings, and the training bearing with the minimum DTW distance to the given test bearing can be selected as the reference bearing of the given test bearing.
3. A parameter optimization method for the FOTP-GM (1, 1) model is proposed to determine the optimal order of time power terms. In this method, the fitting error between the fitted degradation curve and the original degradation trajectory is selected as the evaluation metrics for the training phase, and the distance between the fitted degradation curves of the given testing bearing and corresponding reference training bearing is considered as the selection criteria in the testing phase, which fully considered the difference and similarity of the degradation trajectory of the training bearing and the test bearing
4. A data-driven-based bearing failure threshold setting method is proposed. This method adaptively determines the bearing failure threshold of the given testing using the DTW distance between the given testing and reference training bearing and the life endpoint value of the fitted degradation curve of the reference training bearing, which avoids the blindness of the artificial subjective of the failure threshold setting.

The remainder of this paper is organized as follows.  Section 2 introduces the theoretical background. In Section 3, the failure thresholds setting and RUL prediction methods are proposed and discussed. In Section 4, the experimental procedure and results are presented and discussed. Finally, some conclusions are drawn in Section 5.

## 2. Theoretical Background

### 2.1. Bearing Performance Degradation Characteristics Extraction Based on CWT and CAE

The time-frequency representation provides the joint distribution information of the time domain and frequency domain, and the continuous wavelet transform method is applied to extract the time-frequency distributions of the monitoring bearing signal effectively. The CWT can decompose the given bearing signal into a time-scale plane representation by scaling and shifting the mother wavelet. A mother wavelet *ψ* ∈ *L*^2^(*R*) is usually a function with zero average and finite length, where *L*^2^(*R*) is the space of square-integrable complex functions [45]. The family of time-scale waveforms is obtained by scaling and shifting the mother wavelet as follows:

(1) $$\begin{array}{c} \psi_{a,b}\left(t\right)=\frac{1}{\sqrt{a}}\psi \left(\frac{t-b}{a}\right), \end{array}$$

where *a* > 0 is the scale factor for dilating or contracting the wavelet and *b* is the shifting factor for transitioning the wavelet along the time axis. For the given bearing signal *x*(*t*), the CWT operation decomposes the signal *x*(*t*) into wavelet coefficients according to the following integral:

(2) $$\begin{array}{c} cwt\left(a,b\right)=\frac{1}{\sqrt{a}}\int_{-\infty }^{\infty }x\left(t\right)\psi^{*}\left(\frac{t-b}{a}\right)\text{d}t, \end{array}$$

where *ψ*^*∗*^ is the complex conjugate of mother wavelet *ψ*. The CWT is useful for obtaining the frequency components at different time scales and resolutions. For small scales (*a* > 1), *ψ*_*a*,*b*_(*t*) will be short and of high frequency, while for large scales (*a* < 1), *ψ*_*a*,*b*_(*t*) will be long and of low frequency.

In view of the individual variability of bearing degradation trends, the CAE is used to automatically extract degradation characteristics from bearing monitoring data sets and realize the effective extraction of bearing performance degradation features without prior knowledge of bearing RUL. Compared with the traditional autoencoder, CAE, as an unsupervised deep learning method, uses convolutional operation for the encoding and decoding part instead of slicing and stacking the data, which significantly improves the performance of training parameter optimization and feature extraction [46].

The convolutional network in the CAE encoder encodes the input data into a set of hidden space representations, and then the decoder reconstructs the input data using deconvolution operation. As shown in Figure 1, let *TF*_*i*_ denotes the time-frequency map of the given bearing data *X*_*i*_ at time *i*, where *TF*_*i*_ ∈ *R*^*L*1×*L*1×*D*^, and the *H* represents the potential latent space representations of the given bearing time-frequency data, where *H* ∈ *R*^*L*2×*L*2×*K*^. The *k*th feature map in encoder output *H* can be expressed as follows:

(3) $$\begin{array}{c} H_{k}\left(TF_{i}\right)=\sigma \left(TF_{i}*\omega_{k}+b_{k}\right), \end{array}$$

where *σ*(·) is the nonlinear activation function, *∗* represents 2-D convolution, and *ω*_*k*_ and *b*_*k*_ denote the weights and bias value of the *k*th convolution kernel of the encoder, respectively. Then the *k*th encoded hidden representation can be decoded to reconstruct the input data *TF*_*i*_ using deconvolution operation as follows:

(4) $$\begin{array}{c} {\tilde{TF}}_{i}=\sigma \left(H_{k}*{\tilde{\omega }}_{k}+{\tilde{b}}_{k}\right), \end{array}$$

where ${\tilde{TF}}_{i}\in R^{L1\times L1\times D}$ is the reconstruction of input bearing time-frequency data, ${\tilde{\omega }}_{k}$ is the 2-D deconvolutional filter in the decoder, and ${\tilde{b}}_{k}$ is the bias value of the decoder. During unsupervised pretraining, the loss function of CAE is defined as follows:

(5) $$\begin{array}{c} E={\left\|TF_{i}-{\tilde{TF}}_{i}\right\|}^{2}, \end{array}$$

where *E* denotes the mean-square-error (MSE) distortion between the original input image *TF*_*i*_ and reconstructed image ${\tilde{TF}}_{i}$. Minimizing the loss function *E* can get an optimal hidden space representation of the input bearing time-frequency data *TF*_*i*_, which can be used as a deep feature of bearing performance degradation at that time *i*.

To improve the training efficiency and generalization capability of the CAE network, multiconvolution layers are usually adopted, and each convolutional layer is followed by a batch normalization layer to make sure that the inputs and outputs of each layer have the same amplitude distribution with input data, which make the CAE can use a larger learning rate for training, accelerate the training speed, and overcome the influence of covariance offset.

### 2.2. Bearing Performance Degradation Trajectory Construction Based on SOM

Due to the different sensitivities to track the degradation trend of bearing performance, the multiscale depth representations extracted by CAE cannot reflect the hidden information of bearings in the degradation process in a unified manner, and it is necessary to map such depth features into a unified performance degradation indicator. To obtain an accurate DI curve of the given bearing, the SOM is used to fuse the multiscale depth representations extracted by CAE into a nondimensional DI.

Let *H*_*i*_ denotes the *n*-dimensional hidden representations of the given bearing time-frequency data *TF*_*i*_ output by encoder, *H*_*i*_=(*h*_*i*_^1^, *h*_*i*_^2^,…, *h*_*i*_^*n*^), where *i*=1,2,…, *N*, *N* is the number of bearing training samples. *W*_*j*_=(*w*_*j*_^1^, *w*_*j*_^2^,…, *w*_*j*_^*n*^) is the weights of the *j* th neuron in the SOM network, where *j*=1,2, ⋯, *M*, *M* is the neuron number of the SOM network. The construction process of DI is illustrated as follows:

1. The normalized *H*_1_ is firstly input into the SOM model, and the winning neuron *c* is selected according to the minimum Euclidean distance standard: *H*_1_ − *W*_*c*_=min*H*_1_ − *W*_*j*_. Then the weight vectors, learning rate, and neighborhood radius are updated according to the method mentioned in reference [17].
2. The training samples, *H*_2_ ~ *H*_*N*_, are input into the SOM network in turn to do the same operation, and when all training samples participate in SOM training, one iteration ends. When the iteration times reach the set threshold, the SOM model established by normal feature samples can be obtained.
3. All the historical time-frequency diagrams of the given bearing are input into the trained SOM model, and the DI trajectory can be obtained using the minimum value of Euclidean distance between hidden feature *H*_*t*_ at time *t* and the weight vector *W*:

(6) $$\begin{array}{c} DI\left(t\right)=\min\left\{H_{t}-W_{1},H_{t}-W_{2},\ldots ,H_{t}-W_{M}\right\}. \end{array}$$

The *DI*(*t*) measures the deviation degree of the bearing hidden representations between degradation conditions and the normal condition in kernel space performed by SOM. A higher DI value represents a more severe degeneration in bearing performance.

### 2.3. Similarity Measure of Bearing Degradation Trajectories Based on DTW

Dynamic time warping, which can effectively cluster time series with noise and time distortion, is an effective pattern dissimilarity measurement technique. DTW-based bearing degradation trend matching is a nonlinear regularization method that combines bearing operation time regularization with degradation trajectory distance calculation. It takes the historical degradation curve of the given testing bearing as the reference template, compares the full-life degradation trajectories of the training bearings with the reference template one by one, and finds the training bearing with minimum trajectory distance as the degradation trend matched training bearing of the given test bearing.

The notation *DI*_train_ denotes the full-life degradation trajectory of a training bearing, and the notation *DI*_*test*_ represents the degradation trajectory of a testing bearing, where *DI*_train_ ∈ *R*^1×*N*_train_^ and *DI*_test_ ∈ *R*^1×*N*_test_^. Define a matrix *d* ∈ *R*^*N*_train_×*N*_test_^, where d(*i*, *j*) represents the distance between point *DI*_train_(*i*) and point *DI*_test_(*j*) to find the most fitting path that passes through a number of grid points of this matrix grid, ensuring the final total distance between the two degradation curves is the shortest. Such a path can be expressed as follows:

(7) $$\begin{array}{c} p=\left(p_{1},p_{2},\ldots ,p_{N_{\text{path}}}\right), \end{array}$$

where *p* represents the regularity degree of the two trajectories, *p*_*k*_=(*i*, *j*), 1 ≤ *k* ≤ *N*_path_; 1 ≤ *i* ≤ *N*_train_;  1 ≤ *j* ≤ *N*_test_ and max(*N*_train_, *N*_test_) ≤ *N*_path_ ≤ *N*_train_+*N*_test_. The grid points through which the path passes are the points on which the two sequences are aligned for calculation. To ensure that each point of *DI*_train_ and *DI*_test_ appears in the path *p*, the *i* and *j* in *p*_*k*_=(*i*, *j*) must be monotonically increasing. The obtained regularized path is required to satisfy the shortest distance path rule:

(8) $$\begin{array}{c} D\left(i,j\right)=d\left(i,j\right)+\min\left[D\left(i-1,j\right),D\left(i,j-1\right),\;D\left(i-1,j-1\right)\right], \end{array}$$

where *D*(*i*, *j*) is the cumulative distance of the two sequences from *p*_1_=(1,1) to *p*_*k*_=(*i*, *j*), that is, the sum of the Euclidean distance d(*i*, *j*) that represents the distance between the point *DI*_life_(*i*) and point *DI*_test_(*j*), namely, the cumulative distance of the smallest neighboring element that can reach the point (*i*, *j*). The value of the last point in matrix *D* is the total cumulative distance of the two sequences and can be considered as the similarity of the two sequences.

Bearings with similar degradation trajectories should have a similar degradation pattern. The failure threshold of the reference training bearing with degradation trend matched with the given testing bearing can be used to determine the failure threshold of the given testing bearing.

### 2.4. The Basic Principle of the FOTP-GM (1, 1) Model

The traditional grey model is only suitable for fitting the time series of pure exponential change law, while the performance degradation of rolling bearings is affected by many complex factors, such as steady disturbance, constant speed disturbance, and acceleration disturbance, and its performance degradation trajectory will not strictly follow the pure exponential change law [21]. FOTP-GM (1, 1), as a new model derived from the grey prediction model, can adaptively change the model structure and parameters according to the dynamic changes of the measured sequence to maximize the fitting and prediction accuracy. The discrete form of the FOTP-GM (1, 1) model is defined as follows:

(9) $$\begin{array}{c} \frac{x^{\left(1\right)}\left(t\right)}{dt}+ax^{\left(1\right)}\left(t\right)=\sum_{i=1}^{h}b_{i}t^{h-i}h\geq 1, \end{array}$$

where *a* is the development index,  *b*_*i*_*i*=1,2,…, *h* is the grey actuating quantity, and *h* is termed as the order of time power terms *b*_*i*_*t*^*h*−*i*^.

Based on the given degradation curve *X*^(0)^, a 1-AGO sequence *X*^(1)^ can be generated by the following:

(10) $$\begin{array}{c} x^{\left(1\right)}\left(k\right)=\sum_{i=1}^{k}x^{\left(0\right)}\left(i\right),\;k=1,2,\ldots ,n. \end{array}$$

Then the parameter sequence *a* and *b*_*i*_*i*=1,2,…, *h* of the FOTP-GM (1, 1) model can be estimated by the least-squares method, and the corresponding time response function can be obtained as follows:

(11) $$\begin{array}{c} {\hat{x}}^{\left(1\right)}\left(t\right)=e^{-at}\left(\sum_{i=1}^{h}b_{i}\int t^{h-i}e^{at}\text{d}t+c\right), \end{array}$$

where *c* is a constant that can be optimized to acquire the minimum error of simulation. The reconstructed sequence can be obtained as follows:

(12) $$\begin{array}{c} {\hat{X}}^{\left(0\right)}=\left\{{\hat{x}}^{\left(0\right)}\left(k\right),k\in \mathbb{N},k\geq 1\right\}=\left\{\begin{array}{cc} {\hat{x}}^{\left(0\right)}\left(k\right)={\hat{x}}^{\left(1\right)}\left(k\right)-{\hat{x}}^{\left(1\right)}\left(k-1\right), & k\in N,\;k\geq 2,\\ {\hat{x}}^{\left(0\right)}\left(1\right)=x^{\left(0\right)}\left(1\right). \end{array}\right. \end{array}$$

The structural parameters of the FOTP-GM (1, 1) model can be adjusted adaptively with the dynamic changes of the actual time sequence, which can fit the homogeneous exponential sequence accurately and approximate the nonhomogeneous exponential sequence without error.

## 3. Methodology

Due to the nonlinearity and uncertainty of the bearing degradation process, it is difficult to predict the RUL of the given bearing accurately. The essential step to this problem is to establish a believable and reasonable mathematical model to characterize such a nonlinear degradation process. Based on the theories mentioned in Section 2, the proposed method is shown in Figure 2, which mainly contains four steps: DI trajectory construction, degradation trend matching, optimal order setting of FOTO-GM (1, 1) model, and the RUL prediction with preset failure thresholds.

Firstly, the time-frequency diagrams of the vibration data of the training and testing bearings are input into the CAE network to extract the deep hidden representations, and the degradation trajectories of the training and testing bearings can be generated from such deep hidden representations using the SOM network. Secondly, the trend similarity between the degradation trajectories of the training and testing bearings is evaluated using DTW, and the degradation trend matching results can be determined using the minimum value in DTW distances. Then, the degradation trajectory models of the training and testing bearings can be obtained by applying FOTO-GM (1, 1) model using an order optimization method. Finally, the RUL prediction of the testing bearing can be realized using the preset failure thresholds and fitted degradation curves of testing bearings.

### 3.1. Data-Driven Based Degradation Trajectory Model Construction

An accurate bearing degradation model can reduce the nonlinearity and uncertainty of the bearing RUL prediction. Based on the theories mentioned in Section 2, the proposed data-driven method for bearing degradation trajectory construction and modeling is shown in Figure 3, which can be summed up as four steps as follows.

1. Generating time-frequency diagrams of the given bearing data using equation (2) given in Section 2.1.
2. Extracting the deep hidden features of obtained time-frequency diagrams using the CAE method mentioned in Section 2.1.
3. Mapping the degradation indicator by inputting the normalized depth hidden features into the pretrained SOM network. The DI curve of the given bearing at time *t*, *DI*(*t*), can be obtained using the minimum value of Euclidean distance between hidden feature *H*_*t*_ and the optimized weight vector *W* of the SOM network.
4. Fitting the *DI*(*t*) sequence of the given bearing using the FOTP-GM (1, 1) model with different time power terms orders, then using the method given in Section 3.2 to evaluate the fitting performance and select the optimal time power terms order *h*.

### 3.2. The Order Determining of the Time Power Terms for the Training and Testing Phase

Since the curve reconstructed by the FOTP-GM (1, 1) model is sensitive to the order of time power terms *b*_*i*_*t*^*h*−*i*^. A fitted degradation trajectory model with a suitable *h* can accurately reflect the process of bearing performance degradation. So an appropriate time power terms order is needed to be selected.

The FOTP-GM (1, 1) model is used to fit data points in the historical degradation trajectory of the given bearing and the corresponding fitted time series,*DI*_fitted_, can be described as follows:

(13) $$\begin{array}{c} DI_{\text{fitted}}=\left\{\begin{array}{cc} {\hat{x}}^{\left(0\right)}\left(k\right)=ue^{pk}+qk^{2}+rk+s, & k\in Z,\;k\geq 2,\\ {\hat{x}}^{\left(0\right)}\left(1\right)=x^{\left(0\right)}\left(1\right), \end{array}\right. \end{array}$$

where *u*, *p*, *q*, *r*, and *s* are the fitting parameters.

For the training phase, the fitting performance of different fitting order of time power terms can be expressed as follows:

(14) $$\begin{array}{c} e_{\text{train}}\left(h\right)=\sqrt{\frac{1}{N}\sum_{n=1}^{N}{\left(DI_{\text{train\_fitted}}\left(n\right)-DI_{\text{train}}\left(n\right)\right)}^{2}}, \end{array}$$

where *e*_train represents the root-mean-square value of fitting error between the origin degradation trajectory *DI*_train_ and the fitted degradation curve *DI*_train_fitted_, *h* ∈ *N*^*∗*^ is the order of time power terms, and *N* is the length of the origin degradation trajectory *DI*_life_. The smaller the value of *e*_train, the smaller the fitting error between the fitted curve and the original curve. To prevent overfitting, the *h* corresponding to the trend transition point in the *e*_train curve can be selected as the optimal order of time power terms for the given training bearing.

For the testing phase, the optimal order of time power terms can be determined using the DTW distance between the fitted degradation curves of the given testing bearing and the corresponding reference training bearing with degradation trend matched:

(15) $$\begin{array}{c} e_{\text{test}}\left(h\right)=DT\;W\left(DI_{\text{train\_fitted}},DI_{\text{test\_fitted}}\right), \end{array}$$

where *DI*_train_fitted_ and *DI*_test_fitted_ are the fitted degradation curves of the reference training bearing and the given testing bearing, respectively. The *h* corresponding to the minimum point in the *e*_test curve and making the fitted curve monotonically increasing can be selected as the optimal time power terms order for the given testing bearing.

### 3.3. The Bearing Failure Threshold Setting and RUL Prediction

The discrepancy and similarity of degradation trajectories are considered to determine the failure threshold of the given testing bearing. The degradation trend of the training bearing, which has a similar degradation trend to the given testing bearing, is selected as the reference performance degradation pattern, and the DI value at the life endpoint is considered to set the testing bearing failure threshold. However, the degradation trajectories of training and testing bearings cannot be the same, so the DTW distance between these two curves, which indicates the similarity of the degradation trend, is considered to reduce the difference between these two degradation curves.

Let *DI*_train_ and *DI*_test_fitted_ represent, respectively, the original DI trajectory and the fitted degradation curve reconstructed by the FOTP-GM (1, 1) model of the given reference training bearing, as shown in Figure 4(a). The *DI*_test_ and *DI*_test_fitted_ denote, respectively, the original DI trajectory and the fitted degradation curve reconstructed by the FOTP-GM (1, 1) model of the given testing bearing, as shown in Figure 4(b). The given testing and training bearings have the minimal value of DTW distance showing a similar degradation trend. As shown in Figure 4(e), the value of *DI*_train_fitted_(*N*) at the life endpoint is considered as the failure threshold of the given training bearing. The failure threshold of the given testing bearing with a similar degradation trend to the training bearing can be determined as follows:

(16) $$\begin{array}{c} \text{threshold}=DI_{\text{train\_fitted}}\left(N\right)+DT\;W\left(DI_{\text{train}},DI_{\text{test}}\right). \end{array}$$

The RUL prediction method of rolling bearings based on FOTP-GM (1, 1) can dynamically optimize the model structure according to the performance decline trend of rolling bearings to obtain the smallest simulation error of the original time sequence as much as possible, with higher prediction accuracy and stronger generalization ability.

As shown in Figure 4(e), the specific implementation method of RUL prediction is as follows: firstly, using the historical DI curve of the given testing bearing, *DI*_test_(*m*), (*m*=1,2,…, *M*), to model and solve the parameters with equation (11). Then, the time correspond *DI*_test_fitted_ function can be solved using equation (13), and several points in the future of *DI*_test_fitted_ can be predicted. When the *DI*_test_fitted_ value reaches the preset failure threshold, it is considered that the whole life is reached. Finally, the RUL can be obtained by subtracting the current operation time *T*_*C*_ from the predicted whole life *T*_*p*_, that is,

(17) $$\begin{array}{c} \text{RUL}=T_{p}-T_{c}. \end{array}$$

## 4. Experimental Verification

### 4.1. Case 1: IEEE PHM 2012 Data Challenge

#### 4.1.1. Experimental System and Data Description

The experimental lifecycle data sets of rolling bearings were collected on the PRONOSTIA platform, provided by the FEMTO-ST Institute [43]. This data set was used in the IEEE PHM 2012 Data Challenge for predicting the RUL of bearings. As shown in Figure 5, the experimental platform conducted accelerated degradation tests to collect degradation data of ball bearings until their total failure, in which 17 bearings were tested under 3 different operating conditions, as shown in Table 1. The first 2 bearings of each group were used to train the run-to-failure data set to build prognostics models, and the remaining 11 bearings were truncated and required to predict the RUL accurately. The sampling frequency of the acceleration signal collected by the test bench is 25.6 kHz, and the data acquisition card (NIDAQCard-9174) collects data once every 10 s, with a time of 0.1 s and 2,560 data points.

#### 4.1.2. The Result of DI Curves Construction

The vibration signals collected from faulty bearings usually contain periodic pulses with shapes similar to the Morlet wavelets. Based on the principle that the shape of the selected wavelet should be similar to the mechanical fault signal, the Morlet-based CWT is applied to extract time-frequency features from the raw vibration signal of bearings.

Figure 6 shows the time-frequency diagrams of the bearing training data sets during the run-to-failure experiment, in which the degradation progress is calculated as a percentage of the operation time over the whole lifetime of the bearing. Generally, the lifecycle of bearing can be divided into three stages: normal, degradation, and failure. The normal stage has two phases: run-in state and steady state. The frequency response of a running-in bearing is concentrated in the rotating zone, and the time-frequency diagram becomes clean with time. The time-frequency diagram of a normal bearing is clean with occasional random shocks seen. In the degradation stage, the time-frequency diagram starts to become cluttered, and the frequency response is concentrated in the middle frequency band. When the degradation progress approaches 100%, the time-frequency diagram becomes very cluttered, and the frequency response has amplitude in all frequency bands. The above analysis shows that the time-frequency diagram can show the frequency energy distribution of bearing vibration signals hinting at the development trend of defects in the time-frequency domain, and the time-frequency characteristics of the bearing vibration signals are sensitive to the bearing degradation.

The time-frequency maps of all the tested bearings are input into the CAE model to perform encoding and decoding operations, and the depth hidden characteristics related to bearing performance degradation can be obtained from the output of the convolutional encoder. The specific parameter settings of the three CNN models are shown in Table 2. The size of input time-frequency maps is 128 × 128 × 3. The convolutional encoder has three convolutional layers and three pooling layers. The size of convolutional kernels in the three convolutional layers is 3 × 3, and the stride is 1 × 1. The tiling sizes for the three pooling layers are 4 × 4, 4 × 4, and 2 × 2, respectively. The batch normalization operation is applied to the output of each convolutional layer to make sure that the inputs and outputs of each convolutional layer have the same distribution with input data. The ReLU function is used for the activation function, and the maximum pooling is used for the pooling layer. The padding parameter in both the convolutional and pooling layers is “SAME” to retain the most significant features of the input maps. The convolutional decoder includes six deconvolutional layers, whose parameters of each layer correspond to those of the convolutional encoder. Except for the last deconvolutional layer, the outputs of all the deconvolutional layers are batch normalized, and the activation function is ReLU function with “SAME” padding.

As illustrated in Table 2, the outputs of the convolutional encoder are output by the pooling layer 3, and its size is 4 × 4 × 15, which means that the hidden layer contains 15 feature maps with a size of 4 × 4. These feature maps can be expanded into a fully connected layer with a size of 1 × 240, and the values in this fully connected layer are the depth features of the bearing time-frequency map extracted by the convolutional autoencoder. Taking bearing 1–1 as an example, the dimension of depth features extracted by CAE is 240, and 4 representative features, including Nos. 59, 74, 113, and 125, are selected, and their curves change with the operation time are shown in Figure 7.

Figure 7 shows that the depth features extracted by CAE have a certain trend with time, which is suitable for the prediction analysis of bearing RUL. However, different depth features have different manners of tracking the degradation trend of bearing performance, in which some features increase with time or decrease with time, and some features suddenly change in amplitude at a certain point in operation time. Note that the depth features extracted by CAE cannot uniformly reflect the degradation process, and all the depth features are mapped into a unified DI by SOM. The first 5% normalized feature sets of each bearing are selected as the training data sets of normal bearing to train the SOM model corresponding to each bearing, and the DI curves can be obtained by inputting the normalized feature sets of all the tested bearing into the well-trained SOM model.

Figure 8 shows that the lifecycle degradation trajectories of the bearings under the same working condition show a similar degradation trend with some differences that can be seen, in which the DI values corresponding to the final failure time points are not the same. It can be seen from Figure 9 that the DI curves of test bearings are obviously heterogeneous with different lengths. Due to the difference in data distribution between full-life bearings and test bearings, the degradation trends of bearings under the same working conditions may be different, while the degradation trends of bearings under different working conditions are similar to some extent, so it is difficult to visually determine the full-life bearings with similar degradation trajectories to test bearings. Therefore, it is necessary to match the trend of the degradation trajectory of each bearing and set a reasonable failure threshold for the test bearing by considering the discrepancy and similarity of degradation trajectories of training and testing bearings.

#### 4.1.3. Bearing Degradation Model Construction Using an Optimized Order of Time Power Terms

The fitted degradation curves with different order of time power terms of FOTP-GM (1, 1) have different abilities to predict the bearing RUL. Using the method proposed in Section 3.2, the fitting performance is evaluated by calculating the fitting error between the origin degradation trajectory *DI*_life_ and the fitted degradation curve *DI*_fit_.  Figure 10 shows the degradation model constructed by FOTP-GM (1, 1) with optimal orders of time power terms.

In the fitting error curves of the FOTP-GM (1, 1) model for training bearings, there exists a trend transition point after which the fitting error is getting smaller fluctuation, as shown in Figure 10. The time power terms order corresponding to such trend transition point can be selected as the optimal order of time power terms for the given training bearing. The training bearings have different fitted degradation curves, which illustrates the heterogeneity of the bearing performance decay. The results of the optimal order and the value of the corresponding fitted degradation curves of training bearings at the life endpoint are listed in Table 3.

#### 4.1.4. Failure Threshold Setting of Testing Bearings

To predict the bearing RUL accurately, a reasonable failure threshold for each testing bearing is needed. The similarity matching analysis is performed between the DI curves of testing bearings and the lifecycle degradation trajectories of the training bearings to classify the testing bearing degradation trends based on the degradation trends of training bearing, and the corresponding training bearing degradation model can be selected as the reference degradation model of the selected test bearing. Using the method mentioned in Section 2.3, the similarities between the lifecycle degradation trajectories of the training bearings and the DI curves of testing bearings are illustrated in Table 3.

Based on Tables 3 and 4, the failure thresholds of the testing bearings can be obtained using equation (16) given in Section 3.3 and illustrated in Table 5.

#### 4.1.5. Bearing Remaining Useful Life Prediction

Based on the fitted DI curves and the preset failure thresholds of the test bearings, FOTP-GM (1, 1) model is adopted to predict the RUL of the test bearings using an optimal time power terms order selection method introduced in Section 3.2. The performance of each order of time power terms of the trained model is evaluated quantitatively according to equation (15). Then the RUL of the given testing bearing can be estimated using the optimal fitted degradation curve and the preset failure threshold. For instance, the *e*_test_ curves, the optimal fitted degradation curves, and the RUL prediction results of bearings 1_3, 2_7, and 3_3 are shown in Figure 11.

As shown in Table 6, the optimal order of the FOTP-GM (1, 1) is different for different testing bearings. Table 6 also illustrates the predicted RULs and the error rate of the testing bearings, in which the RUL prediction results of bearings 1_5 and 1_6 are 5,340 s and 4,380 s. However, the given actual RULs of these two bearings are 1,610 s and 1,460 s. The RUL prediction errors of bearings 1_5 and 1_6 are large, which results in poor prediction performance of the proposed method. It seems that the proposed method fails to predict the RULs of these two bearings accurately. However, reference [30] pointed out that bearings 1_5 and 1_6 have their own specificities in the IEEE PHM 2012 prognostic challenge data sets. The data set description document states that “For security reasons, tests were stopped when the amplitude of the vibration signal overpassed 20 g.” However, bearings 1_5 and 1_6 did not meet this requirement. As shown in Figure 12, the waveform of the last sample of bearings 1_3, 1_5, 1_6, and 1_7 are displayed with the amplitude threshold 20 g marked. Figure 12 illustrates that at the end of the test, the vibration peak amplitude of bearings 1_5 and 1_6 are around 10 g and did not overpass the preset failure threshold of 20 g.

To further verify that whether the vibration amplitudes of bearings 1_5 and 1_6 have reached the preset failure threshold, the whole life vibration peak amplitude curves of these two bearings are presented in Figure 13. Figure 13 indicates that the vibration amplitudes of bearings 1_5 and 1_6 did not pass over 20 g during the whole testing process, which means that the given reference RULs of these two bearings are shorter than their real RUL in the case that the failure threshold is set to 20 g. So it is reasonable that the RUL prediction results of the proposed method for bearings 1_5 and 1_6 are longer than the given reference RUL. The error rates of the RUL prediction results of bearings 1_5 and 1_6 are not representative due to the given reference RULs being smaller than their actual RULs.

The performance of the RUL prediction results of testing bearings can be evaluated using three metrics: root-mean-square error (RMSE), symmetric mean absolute percentage error (SMAPE), and scoring function. The RMSE and SMAE are defined as follows:

(18) $$\begin{array}{c} \text{RMSE}=\sqrt{\frac{1}{n}\sum_{i=1}^{n}{\left({\text{actRUL}}_{i}-{\text{RUL}}_{\text{i}}\right)}^{2}},\\ \text{SMAPE}=\frac{1}{n}\overset{n}{\underset{i=1}{\sum }}\frac{2*\left|{\text{actRUL}}_{i}-{\text{RUL}}_{i}\right|}{\left(\left|{\text{actRUL}}_{i}\right|+\left|{\text{RUL}}_{i}\right|\right)}. \end{array}$$

The scoring function has been adopted by many researchers and IEEE PHM 2012 Prognostic Challenge [46]. By considering the different weights of earlier and later prediction results, the scoring function is defined as follows:

(19) $$\begin{array}{c} \left\{\begin{array}{c} E_{i}=\frac{\left({\text{actRUL}}_{i}-{\text{RUL}}_{i}\right)}{{\text{actRUL}}_{i}},\\ A_{i}=\left\{\begin{array}{cc} \exp\left(-\ln\left(0.5\right)\left(\frac{E_{i}}{5}\right)\right), & \text{if }E_{i}\leq 0,\\ \exp\left(+\ln\left(0.5\right)\left(\frac{E_{i}}{20}\right)\right), & \text{if }E_{i}>0, \end{array}\right.\\ \text{Score}=\frac{1}{n-1}\sum_{1}^{n-1}A_{i}, \end{array}\right. \end{array}$$

where *i∈* [1, 11] states for the test bearings defined in Table 1, actRULi and RULi denote the RUL of the bearing estimated by the experimental participants and the actual RUL to be predicted, respectively. *E*_*i*_ is the percent prediction error on testing bearing *i*, and *A*_*i*_ is the score of accuracy of RUL estimates for testing bearing *i*. The Score represents the overall accuracy of testing bearing RUL prediction, and higher value in Score, higher overall RUL prediction accuracy.

To verify the performance of the proposed method, several state-of-the-art RUL prediction methods are compared, including Sutrisno's vibration frequency signature anomaly detection and survival time ratio [13], Hong's combinatorial feature extraction and self-organization mapping [17], Guo's recurrent neural-network-based health indicator [24], Singleton's extended Kalman filter-based method [46], Zhu's multiscale convolutional neural network-based method [22], Cheng's transferable convolutional neural network-based method [29], Mao's deep feature representation and transfer learning [30], and Li's deep adversarial neural networks-based method [33].

Table 7 shows that the proposed method has an outstanding prediction performance. Compared with Sutrisno, Singleton, and Cheng's methods, the prediction RMSE of the proposed method is much smaller. Besides, compared with Mao's method, although the RMSE and score of the proposed method are slightly smaller, the proposed method has the lowest SMAPE value, showing that the proposed prediction model still has better precision. Combined with listed methods, the adaptive failure threshold setting enables the proposed method to predict the bearing RUL accurately under multiple operating conditions.

### 4.2. Case 2: XJTU-SY Bearing Data Sets

#### 4.2.1. Experimental System and Data Description

The experimental lifecycle data sets of rolling bearings provided by the Institute of Design Science and Basic Component at Xi'an Jiaotong University [44] are analyzed to further prove the effectiveness of the proposed method. As shown in Figure 14, the experimental platform consists of an AC motor, a motor speed controller, a rotating shaft, two supporting bearings, a hydraulic loading system, a test bearing, and so on. Two accelerometers (PCB 352C33) are positioned at 90° on the housing of the tested bearing to measure the horizontal and vertical vibrations of the tested bearing. Fifteen rolling element bearings (LDK UER204) were tested under three different operating conditions to collect degradation data of ball bearings until their total failure. As shown in Table 8, the first two bearings of each group were selected to train the run-to-failure data set to build prognostics models, and the remaining nine bearings were truncated and required to predict the RUL accurately. The sampling frequency of the acceleration signal collected by the test bench is 25.6 kHz, and the data acquisition card (LE DT9837) collects data once every minute, with a time of 1.28 s and 32,768 data points.

#### 4.2.2. The Result of DI Curves Construction

The Morlet-based CWT method is applied to obtain the time-frequency diagrams from the vibration data sets of the six training bearings, as shown in Figure 15. Similar to Case 1, the time-frequency map of a normal bearing is clean with occasional random shocks seen. In the degradation stage, the time-frequency diagram starts to become cluttered, and the frequency response is concentrated in the middle frequency band. When the degradation progress approaches 100%, the time-frequency diagram becomes very cluttered, and the frequency response has amplitude in all frequency bands. The above analysis shows that the time-frequency diagram can hint at the development trend of defects in the time-frequency domain, and the time-frequency characteristics of the bearing vibration signals are sensitive to the bearing degradation.

Taking bearing 2_1 as an example, the deep hidden features of its time-frequency diagrams is extracted by the CAE model proposed in Case 1, and four typical feature curves changing with the operation time are shown in Figure 16, including Nos. 57, 94, 168, and 205. Similar to Case 1, Figure 16 indicates that the depth features extracted by CAE have a certain trend with time. However, different depth features have different manners of tracking the degradation trend of bearing performance, in which some features increase with time or decrease with time, and some features suddenly change in amplitude at a certain point in operation time. The SOM method is applied to fuse these depth features into a unified DI to reflect the degradation process uniformly. The first 5% normalized feature sets of each bearing are selected as the training data sets of normal bearing to train the SOM model corresponding to each bearing, and the DI curves can be obtained by inputting the normalized feature sets of all the tested bearing into the pretrained SOM model.

Figures 17 and 18 show that the lifecycle degradation trajectories obtained from the XJTU-SY bearing data sets are obviously heterogeneous with different lengths. Due to the difference in data distribution, the degradation trends of bearings under the same working conditions may be different, while the degradation trends of bearings under different working conditions are similar to some extent, so it is difficult to visually determine the full-life bearings with similar degradation trajectories to test bearings. Therefore, it is necessary to match the trend of the degradation trajectory of each bearing and set a reasonable failure threshold for the given test bearings by considering the discrepancy and similarity of degradation trajectories of training and testing bearings.

#### 4.2.3. Bearing Degradation Model Construction Using an Optimized Order of Time Power terms

The fitted degradation curves with different order of time power terms of FOTP-GM (1, 1) have different abilities to predict the bearing RUL. Using the method proposed in Section 3.2, the fitting performance is evaluated by calculating the fitting error between the origin degradation trajectory *DI*_life_ and the fitted degradation curve *DI*_fit_.  Figure 19 shows the degradation model of training bearings constructed by FOTP-GM (1, 1) with optimal orders of time power terms.

Similar to Case 1, there exists a trend transition point after which the fitting error is getting smaller fluctuation in the fitting error curves of the FOTP-GM (1, 1) model for training bearings, as shown in Figure 19. The time power terms order corresponding to such trend transition point can be selected as the optimal order of time power terms for the given training bearing. The results of the optimal order and the value of the corresponding fitted degradation curves of training bearings at the life endpoint are listed in Table 9.

#### 4.2.4. Failure Threshold Setting of Testing Bearings

To verify the predictive capability of the proposed method, the data sets of testing bearings are segmented with different prediction starting points to perform 10 subtasks, in which the division ratio includes 50%, 55%, 60%, 65%, 70%, 75%, 80%, 85%, 90%, and 95%, as shown in Table 10.

Taking subtask #6 with the division ratio of 75% as an example, the similarity matching analysis is performed between the historical DI trajectories of testing bearings and the lifecycle degradation trajectories of the training bearings to match the testing bearing degradation trends with the degradation trends of training bearing, and the corresponding training bearing degradation model can be selected as the reference degradation model of the selected test bearing. Using the method presented in Section 2.3, the similarities between the lifecycle degradation trajectories of the training bearings and the historical DI curves of testing bearings are illustrated in Table 11.

Based on Tables 9 and 11, the failure thresholds of the testing bearings can be achieved using equation (16) given in Section 3.3 and illustrated in Table 12.

#### 4.2.5. Bearing Remaining Useful Life Prediction

The RUL of the given testing bearing can be estimated using the optimal time power terms order and the preset failure threshold. The RUL prediction results of subtask #6 are listed in Table 13, and for different testing bearings, the optimal order of the FOTP-GM (1, 1) is different.

The predicted whole lives of the testing bearings are shown in Table 14. Due to the different division ratios used to generate the testing samples, the predicted lives of the testing bearings are different. The proposed method can adaptively update the degradation curve fitting model and failure threshold of the given test bearing based on the collected bearing information. As shown in Table 14, the life prediction results get a smaller fluctuation and become more accurate as the volume of testing bearing data increases.

The results of RUL predictions are shown in Figure 20. As can be seen from the figure, the predicted results fluctuate around the actual RUL label values. This preliminarily proves the effectiveness of our proposed method on XJTU-SY data sets. To further illustrate the performance of the proposed method, the RMSE and SMAPE are also utilized as performance evaluation metrics in the RUL prediction of XJTU-SY data sets. The prediction results of the proposed method are compared with the results reported in three published studies, including Huang's deep convolutional neural network-bootstrap integrated method [21], Hu's LSTM predictor trained simultaneously within a generative adversarial network (GAN) architecture [23], Ding's deep subdomain adaptive regression network [32], Li's deep adversarial neural networks-based method [33], and Xiao's trend-reconstruct-based features selection and gated recurrent unit network [47].

Table 15 shows the performance comparison results of the proposed method and five published studies on XJTU-SY data sets. It can be seen that the proposed method achieves a smaller SMAPE value compared with all other methods. Compared with Huang, Hu, Ding, and Li's methods, the proposed method achieves a smaller RMSE value. Compared with Xiao's method, the proposed method has a slightly higher RMSE but has a lower SMAPE. The comparison listed in Table 15 still signifies that the proposed method performs a better performance in the RUL prediction of rolling bearings.

## 5. Conclusions

This paper proposes a new method that involves the difference and the similarity between the degradation trajectories of training and testing bearing to predict the RUL of roller bearings. This method mainly focuses on two aspects of bearing RUL prediction: data-driven based accurate failure threshold setting and optimal mathematical degradation model construction using deep features. From the experimental results, we have the following conclusions:

1. The CAE-based feature extraction method can adaptively extract the deep features associated with the bearing performance degradation. The SOM-based DI construction method can effectively handle the deep features extracted by CAE into a practical degradation indicator.
2. The FOTO-GM (1, 1) model parameter optimization method can determine the optimal fitting order based on the fitting errors. The optimized FOTO-GM (1, 1) method can construct the fitting degradation model of the given bearing based on the degradation information.
3. The failure thresholds setting method based on DTW and optimized FOTO-GM (1, 1) can adaptively adjust the failure threshold of the given bearing according to the accumulation of test bearing information without human intervention.

The proposed bearing RUL prediction model can adaptively update its parameters when new monitoring data are available. The comparison between the experimental results of this method and the existing methods shows that this method can effectively improve the prediction accuracy, reduce the uncertainty of prediction, and has better engineering practicability.

## Figures and Tables

**Figure 1:** Schematic diagram of convolutional autoencoder.

**Figure 2:** Flowchart of proposed bearing RUL predicted method.

**Figure 3:** Building procedure of bearing degradation model using FOTP-GM (1, 1) model.

**Figure 4:** The bearing failure threshold setting and RUL prediction considering the difference and similarity of degradation trajectories.

**Figure 5:** Overview of PRONOSTIA [43] experimental platform.

**Figure 6:** The lifecycle time-frequency plots of the training bearing.

**Figure 7:** The curves of depth characteristics over operation time of bearing 1–1: (a) No. 59, (b) No. 74, (c) No. 113, and (d) No. 125.

**Figure 8:** The lifecycle DI curves of: (a) bearing 1_1, (b) bearing 2_1, (c) bearing 3_1, (d) bearing 1_2, (e) bearing 2_2, and (f) bearing 3_2.

**Figure 9:** The DI curves of testing data sets: (a) bearing 1_3, (b) bearing 1_4, (c) bearing 1_5, (d) bearing 1_6, (e) bearing 1_7, (f) bearing 2_3, (g) bearing 2_4, (h) bearing 2_5, (i) bearing 2_6, (j) bearing 2_7, and (k) bearing 3_3.

**Figure 10:** The fitting error curve and fitted degradation model of: (a) bearing 1_1, (b) bearing 2_1, (c) bearing 3_1, (d) bearing 1_2, (e) bearing 2_2, and (f) bearing 3_2.

**Figure 11:** The DTW distance curves, fitted degradation curves, and RUL prediction results of: (a) bearing 1_3, (b) bearing 2_7, and (c) bearing 3_3.

**Figure 12:** The waveforms of the last sample of: (a) bearing 1_3, (b) bearing 1_5, (c) bearing 1_6, and (d) bearing 1_7.

**Figure 13:** The whole life peak amplitude curves of: (a) bearing 1_5 and (b) bearing 1_6.

**Figure 14:** Overview of XJTU's experimental platform [44].

**Figure 15:** The lifecycle time-frequency plots of the training bearings.

**Figure 16:** The curves of depth characteristics over operation time of bearing 2–1: (a) No. 57, (b) No. 94, (c) No. 168, and (d) No. 205.

**Figure 17:** The lifecycle DI curves of: (a) bearing 1_1, (b) bearing 2_1, (c) bearing 3_1, (d) bearing 1_2, (e) bearing 2_2, and (f) bearing 3_2.

**Figure 18:** The lifecycle DI curves of testing data sets: (a) bearing 1_3, (b) bearing 1_4, (c) bearing 1_5, (d) bearing 2_3, (e) bearing 2_4, (f) bearing 2_5, (g) bearing 3_3, (h) bearing 3_4, and (i) bearing 3_5.

**Figure 19:** The fitting error curve and fitted degradation model of: (a) bearing 1_1, (b) bearing 2_1, (c) bearing 3_1, (d) bearing 1_2, (e) bearing 2_2, and (f) bearing 3_2.

**Figure 20:** The RUL prediction results of 10 subtasks: (a) bearing 1_3, (b) bearing 1_4, (c) bearing 1_5, (d) bearing 2_3, (e) bearing 2_4, (f) bearing 2_5, (g) bearing 3_3, (h) bearing 3_4, and (i) bearing 3_5.

**Table 1:** Data sets of IEEE 2012 PHM prognostic challenge.

Data sets	Operating conditions		
	Condition 1	Condition 2	Condition 3
Speed (RPM)	1,800	1,650	1,500
Load (N)	4,000	4,200	5,000
Training sets	Bearing 1_1	Bearing 2_1	Bearing 3_1
	Bearing 1_2	Bearing 2_2	Bearing 3_2
Testing sets	Bearing 1_3	Bearing 2_3	Bearing 3_3
	Bearing 1_4	Bearing 2_4	
	Bearing 1_5	Bearing 2_5	
	Bearing 1_6	Bearing 2_6	
	Bearing 1_7	Bearing 2_7	

**Table 2:** Specific setting parameters of the convolutional encoder.

Layer	Parameters	Output size	Activation function
Input layer	—	128 × 128 × 3	—
Convolutional layer 1	15 kernels, size: 3 × 3	128 × 128 × 15	ReLU
Pooling layer 1	Size: 4 × 4, stride: 4 × 4	32 × 32 × 15	—
Convolutional layer 2	15 kernels, size: 3 × 3	32 × 32 × 15	ReLU
Pooling layer 2	Size: 4 × 4, stride: 4 × 4	8 × 8 × 15	—
Convolutional layer 3	15 kernels, size: 3 × 3	8 × 8 × 15	ReLU
Pooling layer 3	Size: 2 × 2, stride: 2 × 2	4 × 4 × 15	—
Fully connected layer	240 neurons	1 × 240	—

**Table 3:** The value of fitted degradation curves of training bearings at the life endpoint.

Training bearing	B 1_1	B 1_2	B 2_1	B 2_2	B 3_1	B 3_2
Sample length (10s)	2,803	871	911	797	515	1,637
Optimal order	2	4	6	4	4	4
*DI*_train_fitted_(*N*)	0.5457	0.4368	0.2914	0.5333	0.2659	0.3702

**Table 4:** The DTW distances between *DI*_train_ and *DI*_test_.

Training bearings	Testing bearings										
	B 1_3	B 1_4	B 1_5	B 1_6	B 1_7	B 2_3	B 2_4	B 2_5	B 2_6	B 2_7	B 3_3
B 1_1	0.5591	0.9381	38.5134	18.2890	0.2406	37.5987	0.9118	24.8003	17.2799	1.0701	47.5313
B 1_2	0.9315	0.2254	1.4864	2.7099	1.8439	1.2902	0.4565	4.8017	1.0021	0.6241	0.9382
B 2_1	2.1973	0.9867	0.5670	1.3385	0.2982	0.3149	0.3211	0.3491	0.3925	0.1425	0.1638
B 2_2	0.7220	0.1774	1.8887	2.9778	1.3142	1.3712	0.8598	1.1538	1.2428	0.7570	1.4594
B 3_1	1.8556	1.6527	0.6120	0.7400	0.3929	0.3620	0.5413	0.5899	0.4178	0.2314	0.2649
B 3_2	0.8017	0.5397	1.5497	1.6687	1.1098	1.194	1.0822	1.1779	1.0373	0.6441	1.3180

**Table 5:** The failure threshold setting of the testing bearings.

Threshold setting	Testing bearings										
	B 1_3	B 1_4	B 1_5	B 1_6	B 1_7	B 2_3	B 2_4	B 2_5	B 2_6	B 2_7	B 3_3
Reference bearing	B 1_1	B 2_2	B 2_1	B 3_1	B 1_1	B 2_1	B 2_1	B 2_1	B 3_1	B 2_1	B 2_1
*DI*_train_fitted_(*N*)	0.5457	0.5333	0.2914	0.2659	0.5457	0.2914	0.2914	0.2914	0.2659	0.2914	0.2914
DTW distance	0.5591	0.1774	0.5670	0.7400	0.2406	0.3149	0.32110	0.3491	0.3925	0.1425	0.1638
Failure threshold	1.1048	0.7107	0.81.0059584	1.0059	0.7863	0.6063	0.7579	0.6405	0.6839	0.4339	0.4552

**Table 6:** The RUL prediction results of the testing bearings.

	Testing bearings										
	B 1_3	B 1_4	B 1_5	B 1_6	B 1_7	B 2_3	B 2_4	B 2_5	B 2_6	B 2_7	B 3_3
Optimal order	2	2	8	7	7	5	5	7	6	4	8
Current sample point	1,802	1,139	2,302	2,302	1,502	1,202	612	2,002	572	172	352
Predicted life (10 s)	2,440	1,391	2,836	2,740	2,410	1,940	759	2,314	726	219	430
Predicted RUL (10 s)	638	252	534	438	908	738	147	312	156	47	78
Actual RUL (10 s)	573	339	161	146	757	753	139	309	129	58	82
Error rate (%)	–11.34	12.80	–231.6	–200	–19.95	1.992	–5.755	–0.971	–19.38	18.99	4.878

**Table 7:** The comparison of RUL prediction results of testing bearings.

Methods	RMSE	SMAPE	Score
Sutrisno's method [13]	0.3187	0.3583	0.3066
Singleton's method [14]	0.1161	0.3768	0.2645
Hong's method [17]	0.0907	0.2258	0.3614
Zhu's method [22]	0.0691	0.1549	0.3624
Guo's method [24]	0.0860	0.1910	0.2631
Cheng's method [29]	0.0971	0.2769	0.3035
Mao's method [30]	0.0558	0.2399	0.4285
Li's method [33]	0.0950	0.1516	0.3974
Proposed method	0.0653	0.1373	0.4182

**Table 8:** The description of XJTU-SY bearing data sets.

Data sets	Operating conditions		
	Condition 1	Condition 2	Condition 3
Speed (RPM)	2,100	2,250	2,400
Load (kN)	12	11	10
Training sets	Bearing 1_1	Bearing 2_1	Bearing 3_1
	Bearing 1_2	Bearing 2_2	Bearing 3_2
Testing sets	Bearing 1_3	Bearing 2_3	Bearing 3_3
	Bearing 1_4	Bearing 2_4	Bearing 3_4
	Bearing 1_5	Bearing 2_5	Bearing 3_5

**Table 9:** The value of fitted degradation curves of training bearings at the life endpoint.

Training bearing	B 1_1	B 1_2	B 2_1	B 2_2	B 3_1	B 3_2
Sample length	122	160	491	161	2,538	2,495
Optimal order	7	5	4	5	3	6
*DI*_train_fitted_(*N*)	0.5230	0.6050	0.5892	0.6460	0.6586	0.3708

**Table 10:** The sample size of the inputting testing data sets for 10 subtasks.

Tasks	Division ratio (%)	Percentage of RUL (%)
#1	50	50
#2	55	45
#3	60	40
#4	65	35
#5	70	30
#6	75	25
#7	80	20
#8	85	15
#9	90	10
#10	95	5

**Table 11:** The DTW distances between *DI*_train_ and *DI*_test_ for prediction moment at 75%.

Training bearings	Testing bearings								
	B 1_3	B 1_4	B 1_5	B 2_3	B 2_4	B 2_5	B 3_3	B 3_4	B 3_5
B 1_1	0.3885	0.1917	1.8845	0.5833	0.0317	0.5604	4.4785	5.1261	3.0559
B 1_2	0.0265	0.1847	8.3485	0.0587	0.0337	2.3187	15.6125	16.6287	3.3279
B 2_1	0.2763	1.2976	1.0251	0.5211	0.5866	0.2730	2.5395	2.8445	18.116
B 2_2	0.0414	0.3880	5.2916	0.0689	0.0471	1.1667	11.1385	12.4954	3.45680
B 3_1	0.8931	16.3583	4.5686	0.3993	2.8968	0.98720	8.4642	9.1995	177.3139
B 3_2	0.6146	5.4613	1.1846	1.5713	0.9797	0.5043	2.052	2.3015	134.2678

**Table 12:** The failure threshold setting of the testing bearings for prediction moment at 75%.

Threshold setting	Testing bearings								
	B 1_3	B 1_4	B 1_5	B 2_3	B 2_4	B 2_5	B 3_3	B 3_4	B 3_5
Reference bearing	B 1_2	B 1_2	B 2_1	B 1_2	B 1_1	B 2_1	B 2_1	B 2_1	B 3_1
*DI*_train_fitted_(*N*)	0.5230	0.6050	0.5892	0.6460	0.6586	0.3708	0.5230	0.6050	0.5892
DTW distance	0.0265	0.1847	1.0251	0.0587	0.0317	0.2730	2.0520	2.3015	3.0559
Failure threshold	0.5495	0.7897	1.6143	0.7047	0.6933	0.6438	2.575	2.9065	3.6451

**Table 13:** The RUL prediction results of the testing bearings for prediction moment at 75%.

	Testing bearings										
	B 1_3	B 1_4	B 1_5	B 1_6	B 1_7	B 2_3	B 2_4	B 2_5	B 2_6	B 2_7	B 3_3
Optimal order	2	2	8	7	7	5	5	7	6	4	8
Current sample point	118	91	39	399	31	254	278	1,136	85	118	91
Predicted life (min)	148	118	58	491	43	319	351	1,606	136	148	118
Predicted RUL (min)	30	27	19	92	12	65	73	470	51	30	27

**Table 14:** The predicted lives of the testing bearings for 10 subtasks.

Testing bearings	Tasks									
	50%	55%	60%	65%	70%	75%	80%	85%	90%	95%
B 1_3	155	155	135	134	149	148	152	152	157	157
B 1_4	109	122	96	106	119	118	134	124	126	136
B 1_5	50	65	64	64	60	49	45	55	54	53
B 2_3	447	456	569	534	510	491	437	529	523	521
B 2_4	55	56	49	47	45	43	43	40	39	40
B 2_5	350	342	323	328	305	319	339	334	339	332
B 3_3	380	382	346	350	383	351	395	381	361	353
B 3_4	1,609	1,609	1,591	1,542	1,568	1,606	1,536	1,588	1,518	1,605
B 3_5	132	136	121	119	132	136	123	112	122	118

**Table 15:** The comparison of RUL prediction results of testing bearings.

Methods	RMSE	SMAPE
Huang's method [21]	0.161	0.128
Hu's method [23]	0.238	0.143
Ding method [32]	0.179	0.149
Li's method [33]	0.136	0.144
Xiao's method [47]	0.083	0.109
Proposed method	0.091	0.0833

## Data Availability

The data used to support the findings of this study are included within the article.
